The article "A Novel Intelligent Hybrid Optimized Analytics and Streaming Engine for Medical Big Data" was retracted in 2023. Reasons: signs of a paper mill; compromised peer review; unreliable results or conclusions.

# A Novel Intelligent Hybrid Optimized Analytics and Streaming Engine for Medical Big Data

**DOI:** 10.1155/2022/7120983

**Published:** 2022-03-17

**Authors:** M. Thilagaraj, B. Dwarakanath, V. Pandimurugan, P. Naveen, M. S. Hema, S. Hariharasitaraman, N. Arunkumar, Petchinathan Govindan

**Affiliations:** ^1^Department of Electronics and Instrumentation Engineering, Karpagam College of Engineering, Coimbatore, India; ^2^Department of Information Technology, SRM Institute of Science and Technology, Ramapuram Campus, Bharathi Salai, Ramapuram, Chennai, 600 089 Tamil Nadu, India; ^3^School of Computing Science and Engineering, VIT Bhopal University, Kotri Kalan, Ashta, Near, Indore Road, Bhopal, Madhya Pradesh 466114, India; ^4^Department of Electronics and Communication Engineering, Sri Eshwar College of Engineering, Coimbatore, India; ^5^Anurag University, School of Engineering, Department of Information Technology, Venkatapur, Ghatkesar Rd, Hyderabad, Telangana 500088, India; ^6^Department of Biomedical Engineering, Rathinam Technical Campus, Coimbatore 641021, India; ^7^Department of Electrical and Electronics Technology, Ethiopian Technical University, Addis Ababa, Ethiopia

## Abstract

Medical data processing is exponentially increasing day by day due to the frequent demand for many applications. Healthcare data is one such field, which is dynamically growing day by day. In today's scenario, an enormous amount of sensing devices and data collection units have been employed to generate and collect medical data all over the world. These healthcare devices will result in big real-time data streams. Hence, healthcare-based big data analytics and monitoring have gained hawk-eye importance but needs improvisation. Recently, machine and deep learning algorithms have gained importance to analyze huge amounts of medical data, extract the information, and even predict the future insights of diseases and also cope with the huge volume of data. But applying the learning models to handle big/medical data streams remains to be a challenge among the researchers. This paper proposes the novel deep learning electronic record search engine algorithm (ERSEA) along with firefly optimized long short-term memory (LSTM) model for better data analytics and monitoring. The experimentations have been carried out using Apache Spark using the different medical respiratory data. Finally, the proposed framework results are contrasted with existing models. It shows the accuracy, sensitivity, and specificity like 94%, 93.5%, and 94% for less than 5 GB dataset, and also, more than 5 GB it provides 94%, 92%, and 93% to prove the extraordinary performance of the proposed framework.

## 1. Introduction

The productivity growth enhances during the past few decades such as big data technologies have been spotlighted as a basic fundamental strategy for various innovative aspects on healthcare, public sectors, retailing, and manufacturing [1]. Gartner defined this big data analytics [2] with the three perks that valuable perceptions can be extirpated from the data, made ameliorate decisions from those valuable perceptions, and can be autonomous. Big data streaming constitutes the thumbprint characteristics [3] of rapid speed, real time, and massive volume for various applications which inculcates subsided low latency with hovering throughput distributed messages and parallel processing. Therefore, the evolution of healthcare conventions and research spotlights on big data stream computing for the enhancement in endowments of healthcare services like reduction of cost in prediction and decision-making in real time [4]. The augmentation and utilization of healthcare monitor devices generate patient-related clinical data in real time [5]. The clinical data includes electronic health records, biomedical imaging (“ultrasound, MRI, PET, CT, elastography, EMA, dynamic PET, and hyperpolarised MRI”), sensing data (electroneurogram (ENG), electromyogram (EMG), electrocardiogram (ECG), electroencephalogram (EEG), electrogastrogram (EGG), and phonocardiogram (PCG)), and clinical text mining (natural language processing (NLP)) [6] depicted in Figure 1. Furthermore, the clinical-related data in inconsistency nature expands the repository in idioms of variety, volume, velocity, and veracity. The privileged massive data in healthcare utilized by big data streaming plays a vital role in analytics using many predictions and recommendation systems [7, 8]. The artificial intelligence-based recommendation system [9] with handcrafted autonomous programs based on massive predefined codes was focused by the researchers to solve comprehensible solving problems like chess, even though it is immature to handle the serious complex issues where rules are so hard, to classify the images, object detection, and language translation [10]. Thereby, machine learning came into existence to replace the AI, built by excluding the predefined rules that can work with the very complex datasets [11]. ML based on feature engineering is classified into three categories as “(i) supervised, (ii) unsupervised, and (iii) reinforcement learning.” In supervised learning, the relationship between input and output is labeled as training data, and in unsupervised learning, in contrast, the hidden patterns are identified in the dataset without labeling. Finally, reinforcement learning focuses on the accuracy of the algorithm that enhances with some rewards [12]. These algorithm-based ML approaches generate good results on the well-organized structured data; however, it felt challenges on facing the unstructured domain [10]. To overcome these issues with ML approaches to handle the big data with complex structures, there arose a deep learning (DL) concept that relies on artificial neural networks (ANN). Deep learning-based ANN uses many layers to probe more complicated nonlinear patterns and matriculate meaningful relationships within the big data, by excluding the requirement of feature engineering [11]. Therefore, healthcare adopting this big data streaming using deep learning often outperforms the ML approaches [12] and generates revolutionary results by excluding the noise and being robust to the variability in divergent schemes. Recent exemplary use of Google Flu Trends based on deep learning networks [13] to analyze the MRI medical image predicts more than the clinicians in terms of high accuracy, high quality, and better efficiency. In the medical system, the applications based on deep learning algorithm are inclusive of “convolution neural network (CNN), recurrent neural network (RNN), deep belief network (DBN), deep neural network (DNN), and generative adversarial network (GAN)” [14]. But still, these deep learning models require more computational overhead which makes them unsuitable for effective data analytics and streaming.

## 2. Scope of the Research

The proposed research is focused on the integration of artificial intelligence for better analytics of big healthcare data and streaming. In this study, the hybrid deep learning model is integrated with the firefly optimization for reduced latency and high throughput. The extensive experimentations have been carried out using electronic health record (EHR) medical data and performance metrics such as accuracy, latency, and throughput that are calculated.

## 3. Related Works

Yamashita et al. [15] proposed the CNN architecture for radiology through backpropagation such as “convolution layers, pooling layers, and fully connected layers.” In this work, the overfitting problem faced by CNN is eliminated. 3D multiview uses the dataset of 1007 chest radiographs. Therefore, the experimentation results reveal that the proposed CNN-based model predicts the presence and classifies the radiology reports with accuracy. Humayun et al. [16] propounded a novel detection of abnormal heart sound using CNN by the front-end bandpass filters within the network that utilizes the time-convolution (tConv) layers. The filters enhance the learning process. The experimentation done with the PhysioNet/CinC 2016 dataset on a balanced 4-fold cross-validation generates the enhanced overall accuracy with the improvement over the baseline. Ismail et al. [17] propounded the abnormality in the prediction of disease using the CNN model for the unstructured EHR. Since CNN uses many layers, the full memory was utilized by the fully connected network structure. To resolve this problem in CNN, the propounded method uses the Pearson correlation coefficient and regular pattern behavior had two layers. The first layer utilizes the health-related attributes, and the second layer analyzes the correlation coefficient and then classifies the positive and negative health factors. Thus, the results obtained are “obesity, high blood pressure, and diabetes.” The result analysis is highly accurate and has a low computational cost because the experimentation incorporates “the real-time health examinations of 10,806 citizens that respond to a health survey with 768 items as 4,759,777 records.” Asemi et al. used fuzzy multicriteria decision-making (MCDM) which is a human judgment-based method for weighting of RSs' properties. Human judgment is associated with uncertainty and gray information [18]. Choi et al. [19] explored the initial diagnosis of heart failure focus on improving the prediction model using deep learning-based model temporal relations. RNN inherits the gated recurrent units to prognose the relations among time-stamped events. Thus, the experimentation was carried out with “3884 incident HF cases and 28,903 controls from primary healthcare-related patients” which enhances the performance in the explored model for the detection of heart failure. Khodabakhshi et al. [20] introduced RNN-based dynamic characterization model for lung sounds. The propounded attractor RNN uses the tool named “Recurrent Quantification Analysis” (RQA) to extract the complex system's nature. The evaluation uses the “27 patients that endure COPD, 31 asthma groups aged within 25–55 years, and 25 healthy persons from 20 to 40 years of age who are nonsmokers with no history of serious pulmonary disorders.” The effectiveness of the propounded model produces the best classification accuracy with the adoption of features of RQA. Maragatham et al. [14] introduce the LSTM-based big data model to predict heart failure. The author builds the model with the use of conventional predictive temporal model LSTM and connected to longitudinal time stepped EHR. SiLU and tanh are the activation functions utilized in this framework. Thus, the results from the experimentation carried out with the “arbitrary samples of 365,446 patients, incident 4289 cases of heart failure, and 30,249 patient controls” were used. It is correlated with the conventional deep learning approaches which showed the better performance in detecting heart failure. Sarker et al. presented the structured and comprehensive view on DL techniques including a taxonomy considering various types of real-world tasks like supervised or unsupervised [21]. Garehbaghi et al. performed the structural risk evaluation relay on the “deep neural network” (DNN). Heart sound signals were analyzed by the designed classifier for the identification of heart disease. The outcome shows better performance in terms of structural risk. Chen et al. [22] explore the novel method to predict drug synergy based on a deep belief network. The author explores by using datasets provided by the “2015 DREAM competition.” The outcome shows better performance in predicting drug synergy. Emami et al. [23] presented generating brain synCTs that incorporate generative adversarial networks. The proposed CNN classifier is utilized to classify the input image into real and synthetic. Performance evaluation is done with the help of a 5-fold cross-validation process. GAN performance was correlated to CNN based on “mean absolute error (MAE), structural similarity index (SSIM), and peak signal-to-noise ratio (PSNR)” metrics between the synCT and CT images. Thus, the results obtained are a strong potential to treat near to the real-time treatment in the brain. San et al. [24] developed a DNN-based intelligent diagnostics system for the prediction of hypoglycemia. This model gives a superior classification process on unprocessed data. For the evaluation, this work used 15 children data with type 1 diabetes. When compared with other methodologies, the proposed framework provides better classification performance and the different surveys are shown in Table 1.

## 4. Apache Spark Engine: An Overview

Apache Spark is a well-known big data processing environment that significantly supports hybrid frameworks. A hybrid framework can support both batch and stream processing. The Spark engine is very similar to Hadoop MapReduce engine, but it outperforms in terms of performance because of its full-time computation capacity. It also runs in standalone mode or combined with Hadoop to change the MapReduce engine.  Table 2 lists the features of Spark layers.

The proposed architecture is formulated by deploying the new hybrid deep learning model to analyze the huge data with greater performance. The proposed model induces the modification in the traditional Spark engine which can be used for the diagnosis of different body abnormalities from the different sources of data.

### 4.1. Proposed Methodology

### 4.2. System Overview

Figure 2 shows the proposed architecture for the hybrid deep learning model to analyze in this section; the proposed intelligent hybrid framework and Apache Spark engine model are explained to improve the performance of big data analytics and streaming in healthcare. In this architecture, the proposed framework is divided into three important phases: streaming layers, prediction layers using the hybrid deep learning model, and output layers. In the first phase, electronic health records of the different patients are then streamed using the Spark streaming layers. These input records consist of different heart abnormalities with different patient IDs. In the second phase, these data are streamed through Spark engine, which is then fed as the input data vectors to the proposed learning model. Since the health records consist of both numerical and string values, data are preprocessed and given as the inputs to the optimized learning mode layer. These layers predict the heart abnormalities such as cardiac arrhythmias and store them in the output layers which can be used for further monitoring. The complete architecture is implemented under the Spark engine.

### 4.3. Healthcare Data Collection

In this layer, data were collected from large databases. The proposed architecture uses electronic health record (EHR) datasets from MIMIC (Medical Information Mart for Intensive Care).

### 4.4. Streaming Layers

The proposed architecture uses Spark's streaming layers to stream the data for further diagnosis. To perform the streaming analysis, the fast scheduling process of Apache Spark is used in the proposed architecture. The data received from the different sources are transformed into minibatches for achieving high-speed streaming.

### 4.5. Hybrid Learning Models

This section discusses the new hybrid model to predict the abnormalities in the EHR of patients. Even though Spark ML offers a variety of learning models for analyzing the different data, it eventually fails in achieving the highest performance which is mandatory for an effective diagnosis. Hence, the proposed hybrid framework used the optimized deep learning model for the prediction of heart abnormalities from the electronic health records of the patients.

#### 4.5.1. Recurrent Neural Networks (RNN)

RNN is a neural network that is specialized to process the sequence of data. Generally, RNN is designed to process the time series data and big data analytics because of its remembrance function and encoding capacity of historical data within ms. In this method, direct graphs can be generated by nodes with their sequences. It uses an internal memory state for data processing. This method significantly used the past data to predict the future values. For the real-time analysis, the RNN may not be suitable because if the intermediate time between past and future data is relatively large, this method cannot remember the past data in an efficient way which is called the disappearing gradient problem [27, 28]. To alleviate this problem, RNN performance has been improved with the introduction of the LSTM network.

#### 4.5.2. LSTM (Long Short-Term Memory)

LSTM is an updated version of an RNN, and it is effectively utilized for different applications because of its flexible nature in memory and huge database handling capacity. The LSTM network is demonstrated in Figure 3.

The proposed hybrid framework incorporates LSTM and firefly optimizer. The LSTM framework has 3 different units called “input gate, forget gate, output gate, and cell input.” It is a memory-based NN framework, and it can remember past values in efficient manner.

Let *x*_*t*_, the unseen layer output is “*h*_*t*_” and its former output is “*h*_*t*−1_”; the cell input state is “*C*_*t*_”; the cell output state is “*G*_*t*_” and its former state is “*G*_*t*−1_”; the three gates' states are *j*_*t*_, *T*_*f*_, and *T*_0_. The formation of LSTM resembles that both “*G*_*t*_ and *h*_*t*_” are communicated to the next neural network in RNN. To calculate *G*_*t*_ and *h*_*t*_, we use the following equations.

(1) $$\begin{array}{c} I\cdot G:j_{t}=\theta \left(G_{l}^{i}\cdot O_{t}+G_{h}^{i}\cdot e_{t-1}+s_{i}\right),\\ F\cdot G:T_{f}=\theta \left(G_{l}^{f}\cdot O_{t}+G_{h}^{f}\cdot e_{t-1}+s_{f}\right),\\ O\cdot G:T_{o}=\theta \;\left(G_{l}^{0}\cdot O_{t}+G_{h}^{o}\cdot e_{t-1}+s_{o}\right),\\ C\cdot I:\tilde{T_{C}}=\tanh\left(G_{l}^{C}\cdot O_{t}+G_{h}^{C}\cdot e_{t-1}+s_{C}\right), \end{array}$$

where *G*_*l*_^0^, *G*_*l*_^*f*^, *G*_*l*_^*i*^, *G*_*l*_^*C*^ are “weight matrices between input gates and output layers” and *G*_*h*_^*i*^, *G*_*h*_^*f*^, *G*_*h*_^*o*^, *G*_*h*_^*C*^ are “weight conditions generated between hidden and input layers”.

*s*_*i*_, *s*_*f*_, *s*_*o*_, *s*_*C*_ are “bias vectors.”

tanh is the hyperbolic function.

The cell output state is determined as follows:

(2) $$\begin{array}{c} T_{C}=k_{t}*\tilde{T_{C}}+T_{f}*T_{t-1},\\ e_{t}=T_{o}*\tanh\left(T_{C}\right). \end{array}$$

The above equation is utilized to obtain the final output score.

#### 4.5.3. Motivation behind the Proposed Model

LSTM exhibits computational overhead when handling larger datasets such as electronic health records (EHR). California health and human service dataset is used for the analytics and streaming engine for big data.  Figure 4 is the complete structure of LSTM training network. LSTM cells consist of dense fully connected layers for effective training. These dense layers are trained by hyperparameters such as bias weights, hidden layers, epochs, and learning rates. As the datasets increase, computational complexity in tuning the hyperparameters increases which result in performance degradation. This creates an impact on the poor diagnosis rate. To overcome this drawback, a new intelligent model is required to predict the heart disease categories. The proposed hybrid framework gives a fine solution for the above-mentioned drawback when the firefly algorithm is integrated with the LSTM framework.

#### 4.5.4. Firefly Swarm Optimization

Firefly algorithm is also known as the family of swarm intelligence algorithms, and it is developed by Yang [27]. These fireflies generally flash their lights in the sky during summer night times. The meaning of flashing lights is either to make attention of matting partner or defend from the enemies [21]. In the firefly algorithm, the value intensity of light is directly corresponding to the fitness value. The upcoming three assumptions are the motivation behind developing a working principle of the algorithm and they are given as follows.

1. All fireflies are assumed to be unisex, and attraction happened among them regardless of their sex
2. Attractiveness is relatively proportional to the brightness of fireflies, and it reduces as the distance increases between them
3. The brightness or the light intensity is computed by the feasible solutions of the objective function

From the assumptions, it is very clear that the firefly intensity *I*(*r*) is inversely proportional to distance (*r*). If the distance increased, the light gets absorbed by the air and vice versa. Let *y* be light absorption; the intensity of light *I*(*r*) concerning distance *r* is given by the following equations.

(3) $$\begin{array}{c} I\left(r\right)=I_{0}e^{-yr2}, \end{array}$$

where *I*_0_ is the initial intensity at the source, and then, *β* (attractiveness parameter) is given as follows:

(4) $$\begin{array}{c} \beta \left(r\right)=\beta_{0}e^{-yr2}. \end{array}$$

*β*_0_ is the attractive parameter at initial distance zero.

Based on the behavioral rule, the firefly positions are determined which are given in the equation below.

(5) $$\begin{array}{c} x_{i+1}=x_{i}+\beta \left(r\left(i,j\right)\right)\left(xj-xi\right)+AE, \end{array}$$

where “ *A* is the randomization factor, *E* is the random number vector derived from the Gaussian distribution, *x*_*i*_ is the *i*^th^ position of the firefly, and *x*_*i*+1_ is the value of attraction.”

#### 4.5.5. Firefly Optimized LSTM Networks

LSTM exhibits less performance when handling big datasets. Normally, the larger datasets require more memory which leads to computational complexity. Motivated by this drawback, the proposed training employs firefly swarm optimized LSTM whose hyperparameters such as epochs and hidden layers are optimized to obtain better performance when compared with the LSTM model. The high diagnosis prediction is kept as the global best function (Gbest). The mathematical expression for the proposed fitness function is given by equation (7). Initially, these hyperparameters are selected randomly and passed to the LSTM training network. For each iteration, hyperparameters are calculated by using equations (3), (4), and (5). The iteration stops when the fitness function matches equation (7). The working mechanism of the proposed architecture is presented in Figure 5 and Algorithm 1.

(6) $$\begin{array}{c} \text{Gbest Function}:\mathrm{Max}\left(\text{Accuracy}\right). \end{array}$$

The working mechanism of the firefly optimized LSTM is given in electronic record search engine algorithm (ERSEA).

### 4.6. Output Storage Layers

After the prediction of the abnormalities in the EHR, the diagnosed data are then stored in the server for further processing and monitoring.

## 5. Results and Discussion

### 5.1. Experimentation Details

The proposed network is implemented in Python API Libraries interfaced with local server, which runs on Windows PC10 pro with i9 CPU, 16 GB NVIDIA Geo-force GPU, 16 GB RAM, and 2.5 GHz. For the experimentation, the proposed framework used the “electronic health record” (EHR) data from a real-time environment to predict abnormal heart diseases. Initially, the 4-year heart disease patient data are extracted first. There are 2 parts in the dataset (part A and part B). The first part set has 5000 heart patient data. The second part has 15000 patients who do not have any heart disease.

### 5.2. Performance Metrics and Evaluation

To prove the extraordinary performance of the proposed hybrid framework, the performance metrics such as accuracy, specificity, and sensitivity are calculated. The mathematical expression for the performance metrics is given

(7) $$\begin{array}{c} \text{Accuracy}=\frac{\text{DR}}{\text{TNI}}\times 100, \end{array}$$

(8) $$\begin{array}{c} \text{Sensitivity}=\frac{\text{TP}}{\text{TP}+\text{TN}}\times 100, \end{array}$$

(9) $$\begin{array}{c} \text{Specificity}=\frac{\text{TN}}{\text{TP}+\text{TN}}\times 100, \end{array}$$

where “TP and TN represent true positive and true negative values and DR and TNI represent number of detected results and total number of iterations.”

Figures 6–9 show the performance of the proposed algorithm with the increased number of datasets and dropout ratio. The dropout plays an important role in maintaining the optimum performance during training and validation [6]. From the above figures, it is clear that the proposed algorithm shows the optimum performance between 98.6% and 99% accuracy though the datasets and dropouts are increased linearly. Hence, this proves that the firefly optimized hyperparameters play an important role in streaming the larger datasets. Furthermore, we have proved the efficiency of the proposed architecture; we have compared the other state of the art of learning algorithms such as “long short-term memory (LSTM, without optimization), support vector machines (SVM), naïve Bayes (NB), *K*-nearest neighborhood (KNN), and deep neural network (DNN).” The evaluation is carried out using the different sizes of medical data [29, 30].

Tables 3 and 4 illustrate the performance metrics of the proposed algorithm for the different data sizes. For the 5 GB data, state-of-the-art learning models have performance than the proposed architecture. It is found that the proposed architecture has produced 92.5% accuracy and proves that it can be used for better prediction [31]. From Table 3, it is found that the other learning models have produced considerably less performance than the proposed architecture when the volume of data increases. Nearly 20% drop in performance is found in other learning models whereas only 2% drop is found in the proposed architecture. Hence, the proposed architecture finds its suitable place in the prediction and diagnosis process. To analyze the overall performance of the proposed streaming engine, we have calculated the parameters such as “throughput (*T*), latency (*L*), and network usage (*N*).”

Figure 10 shows the proposed architecture throughput analysis. From Figure 10, it is clear that the proposed architecture has shown the 98% throughput for the different iterations. Furthermore, the computational latency analysis has been calculated and compared with the traditional streaming engine (Spark engine ML). It is found from Figure 11 that computational latency has reduced to 50% in the proposed architecture than the existing model. Since the proposed hybrid model uses the optimized LSTM for the prediction of heart abnormality, time computation is reduced even to 50% when compared with the other learning models in Spark.

## 6. Conclusion and Future Scope

In this work, we emphasized the usage of an optimized deep learning algorithm in an Apache streaming engine suitable for healthcare data analytics. This integration is the first of its kind and proves an efficient role in the streaming-only diagnosis process. The proposed deep learning architecture has produced 94% prediction accuracy and also consumes only 50% of computational latency and maintains 98% throughput. The main contribution of this research is that we found a way to deploy the high-performance deep learning model in the Spark streaming engine to diagnose the heart abnormalities from the EHR data with low latency and high throughput. Handling huge data is a very hectic job for database administrators in terms of analytics, classification, etc., so this proposed stream engine and its algorithm are helpful to the data analysis part in terms of throughput, latency, and specificity. Though the proposed algorithm has produced 94%, performance still needs its improvisation. Also, we would like to find a method to deploy the learning model to handle the heterogeneous medical data. For future scope, we will apply the same data streaming engine in the Parkinson datasets and try to identify the early detection and prevention method for better healthcare management.

## Figures and Tables

**Figure 1:** Big healthcare data sources.

**Figure 2:** Overall framework for the proposed architecture.

**Figure 3:** LSTM structure.

**Figure 4:** LSTM training networks.

**Figure 5:** Working flowchart for the proposed firefly optimized LSTM for big EHR analysis.

**Figure 6:** Validation curves for the proposed ERSEA for increased number of datasets at dropout = 0.2.

**Figure 7:** Validation curves for the proposed ERSEA for increased number of datasets at dropout = 0.4.

**Figure 8:** Validation curves for the proposed ERSEA for increased number of datasets at dropout = 0.6.

**Figure 9:** Validation curves for the proposed ERSEA for increased number of datasets at dropout = 0.8.

**Figure 10:** Throughput analysis for the proposed DL-based streaming architecture for different volumes of data.

**Figure 11:** Computational latency analysis for the proposed ERSEA-based Spark architecture and traditional streaming architecture.

**Algorithm 1:** Electronic record search engine algorithm.

**Table 1:** Different surveys on medical big data analytic methods with its limitations.

S. no.	Author name and year	Model	Recent application in healthcare	Accuracy	Limitation
1	Yamashita et al. (2018)	CNN	Radiology [15]	99.3% confidence	Need lots of labeled data for classification
2	Humayun et al. (2018)		To detect the abnormal heart sound [16]	Cross-fold Macc of 87.10, an absolute improvement of 9.54% over the baseline CNN system	
3	Ismail et al. (2020)		Health model for regular health factor analysis [25]	Accuracy reaches 95.60%	Only two layers are used to classify the positive and negative correlated factors
4	Choi et al. (2017)	RNN	To detect the onset of heart failure [17]	The AUC for the RNN model increased to 0.883	Require a massive volume of datasets Have various problems due to gradient vanishing
5	Khodabakhshi et al. (2018)		To classify the abnormalities in the lungs [19]	Classification accuracy of 91%	
6	Maragatham et al. (2019)		Prediction of heart failure in big data [14]	0.894 AUC	Delineates the time taken for the training of two diverse LSTM models
7	Gharehbaghi et al. (2018)	DNN	Phonocardiography [20]	Accuracy reaches 92.60%	The learning process is too slow
8	Chen et al. (2018)	DBN	To detect type 1 diabetes [26]	71.5%, recall of 60.2%, and *F* score of 65.4%	The training process is computationally expensive
9	Seeliger et al. (2018)	GAN	Reconstructing natural images from brain activity [22]	72.2% correct identifications	Hard to learn to generate discrete data
10	Emami et al. (2018)		Generating synthetic brain CTs [23]	PSNR was 26.6 ± 1.2 and SSIM was 0.83 ± 0.03	Very hard to train
11	San et al. (2016)	DBN	To detect the hypoglycemic episodes in children with type 1 diabetes [24]	Sensitivity = 80% Specificity = 50%	The initialization process makes expensive computational overhead

**Table 2:** Spark engines' features and its functionalities.

Sl. no.	Spark features	Functionalities
1	Spark SQL	Formerly known as Shark. Spark SQL is a distributed framework that works different categories of data.
2	Spark streaming layers	These layers are used for an effective real-time streaming.
3	Spark ML	This module in Spark provides scalable machine learning algorithms for big data analytics. Moreover, it can be programmed either using Python or Java.
4	Spark R	It is computational R programming packages used for data analytics.
5	GraphX	It is a computational tool used for creating discrete graphs for various data.
6	SparkCore	It is the top core of Spark in which the models are deployed.

**Table 3:** Performance metrics of the different algorithms with the data size of 5 GB.

Algorithms	Performance metrics (%)		
	Accuracy (%)	Sensitivity (%)	Specificity (%)
SVM	88%	85%	84.5%
NB	82%	81.5%	80%
KNN	83%	80%	78%
DNN	87.4%	86.5%	77%
LSTM	89%	88.5%	88%
Proposed ERSEA	94%	93.5%	94%

**Table 4:** Performance metrics of the different algorithms with the data size greater than 5 GB.

Algorithms	Performance metrics (%)		
	Accuracy (%)	Sensitivity (%)	Specificity (%)
SVM	76%	75%	74%
NB	70%	69%	70%
KNN	74%	68%	69%
DNN	73%	67%	72%
LSTM	79%	78.5%	77%
Proposed ERSEA	94%	92%	93%

## Data Availability

The data used to support the findings of this study are available from the corresponding author upon request.
